This article has been retracted.

# HDAC2 Induces DNA Methyltransferase DNMT3B Expression to Regulate the Wnt Signaling Pathway and Thus Promotes Glioma Development and Progression

**DOI:** 10.1155/2022/1948766

**Published:** 2022-10-11

**Authors:** Xing Ren, Zhan Jiang, Ke Xu

**Affiliations:** Department of Oncology, Radiotherapy Center, Chongqing General Hospital, Chongqing, China

## Abstract

**Purpose:**

To investigate the role and molecular mechanism of HDAC2 in glioma.

**Methods:**

GSE16011, GSE31262, and GSE90598 datasets were used to identify co-expressed genes, GO analysis, and KEGG analysis to identify gene enrichment pathways, and PPI networks were constructed to identify gene interrelationships. HDAC2 enrichment on DNMT3B promoter and DNMT3B enrichment on Bcl2 CpG island was detected by a ChIP assay. The expression, prognosis, and hierarchical distribution of HDAC2, DNMT3B, and Bcl2 were examined in the CGGA database, and the correlation between HDAC2 and DNMT3B, Bcl2, and DNMT3B and Bcl2 was assessed.

**Results:**

The HDAC2-DNMT3B-Bcl2 axis is differentially expressed and interacts in gliomas. HDAC2 activates the transcriptional activity of DNMT3B, and DNMT3B inhibits the expression of Bcl2. HDAC2 and DNMT3B are highly expressed in gliomas and have a poor prognosis, while Bcl2 is lowly expressed in gliomas and has a good prognosis.

**Conclusion:**

HDAC2 promotes DNMT3B transcriptional repression of Bcl2 expression and Wnt pathway activity, thereby activating glioma cell activity in vitro and in vivo.

## 1. Introduction

Glioma is a common neurosurgical malignancy with an annual incidence of approximately 3–8 per 100,000 and 30,000 deaths per year. Like other tumors, glioma is caused by genetic and environmental carcinogenic factors. Gliomas are initially undetectable with no apparent symptoms, and as they increase in size or become cystic, symptoms of increased intracranial pressure or cerebrovascular compression such as localized epilepsy appear. When glioma is diagnosed, there are limitations to various treatments due to the specificity of its location, and it cannot be cured entirely, which is highly harmful to human beings. The specific treatment modalities for glioma are surgery, radiation, and chemotherapy. Although surgery has made some progress [1], it is challenging to eradicate glioma because of its aggressiveness and high recurrence rate; radiotherapy is not sensitive to most glioma tumors, and some sensitizers need to be added to assist in treatment. Although traditional chemotherapy is not as fast as surgery and radiotherapy, chemotherapy is still essential. It plays a vital role in glioma recurrence and the killing of residual tumor cells. Studies have shown that ACNU combined with TMZ is often used as adjuvant therapy after surgery and radiotherapy and is effective in preventing glioma recurrence after surgery. [2, 3]. However, the biggest problem facing chemotherapy for glioma is the increase in drug resistance, which is why glioma is challenging to cure, making it one of the worst prognoses among systemic tumor diseases [4]. Therefore, exploring the causes of chemotherapy resistance in glioma patients and trying to find drug resistance targets are of profound significance for glioma prognosis. Numerous studies have shown that histone deacetylase HDAC2 appears to be highly expressed in multiple types of cancer cells. For example, a study of tissue sections from clinical prostate cancer patients revealed that HDAC2 was differentially expressed in different grades of prostate cancer tissues, with higher expression with increasing progression [5]. A study of sections from patients with squamous laryngeal carcinoma revealed that HDAC2 expression was significantly higher in the cancer site than that in the paracancerous tissue, and the survival rate of patients with low expression HDAC2 laryngeal squamous cell carcinoma was high under the same radiotherapy conditions [6]. This shows that the expression of HDAC2 is closely related to the grade of tumor progression, patient survival rate, and drug resistance. Numerous studies have demonstrated HDAC2 overexpression involving transcriptional processes of tumor-related genes such as oncogenes. Some researchers further investigated the relationship between HDAC2 and glioma [7] and found that HDAC2 expression was significantly higher in glioma multidrug-resistant cell lines than that in chemotherapy drug-sensitive lines. HDAC2 belongs to class I HDACs. Based on homology analysis, HDACs were classified into four categories: class I HDACs mainly include HDAC2, 2, 3, 8; class II consists of HDAC4, 5. HDACs are mainly composed of HDAC4, 5, 6, 7, 9, 10. Class III, the silent information regulator 2-related enzyme class, is an NAD + -dependent class of enzymes [8]; class IV HDACs occupy a separate class because they are different from classes I and II, mainly including HDAC21. HDACs are modified when the ATGC arrangement order of DNA HDAC2, as one of the more critical HDACs, has become a keen focus of researchers. HDAC2 mainly regulates histone and some nonhistone modifications. Rampalli et al. [9, 10] investigators found that SMAR1-related proteins in breast cancer are associated with HDAC2 by recruitment of HDAC2 Sin3 and retinoblastoma pocket proteins and inhibited the effects of cyclinD1 on cell cycle aspects by deacetylating the upstream region of cyclinD1 promoter on cyclin and found that the mechanism of action of oncogene SMAR1 is closely related to HDAC2.

The effect of HDAC2 expression on the morbidity trend and prognostic factors of prostate cancer patients was investigated. The deterioration grade of such cancer was proportional to HDAC2 expression. The high expression of HDAC2 in ERG (ETS-related gene) negative tumor cells is closely related to the gene fusion of TMPRSS2-ERG, expression of ERG, and deletion of PTEN, 5q, and 6q. The prognostic impact of HDAC2 is not dependent on established clinicopathological parameters and is expected to be a clinical, biochemical indicator for determining the risk grade of prostate cancer [11]. Aghdassi et al. [12] also found that invasive pancreatic cancer spread and metastasis were associated with the downregulation of E-calcine mucin, which is regulated by deacetylases 1 and 2. Overexpression of deacetylases 1 and 2 can reduce the amount of E-calcine mucin, allowing tumor cells to shuttle through the basement membrane to invade surrounding paracancerous tissues, resulting in enhanced tumor cell invasion and migration.

In contrast, HDACIs (histone deacetylase inhibitors) can inhibit the activity of some HDACs and therefore reduce the migratory force of tumor cells. Kumagai et al. [13, 14] found that in addition to E-calcine mucin, other anticancer factors such as retinoic acid receptor RAR*α*, cycle regulator p21/WAF1, and transcription factor C/EBP*α* are also involved in HDACI-induced growth inhibition in pancreatic cancer. HDACIs, such as valproate (VPA) in combination with temozolomide (TMZ), a classical chemotherapeutic agent for glioma, can significantly increase E-calcine mucin expression in lung cancer in vitro experiments and enhance the efficacy of chemotherapeutic agents by enhancing antitumor treatment [15]. Amaravadi et al. [16] found that HDAC2 inhibitor TSA could enhance the expression of mRNA for the 5-hydroxytryptamine transporter (5-HTT) in HepG2 and THP-1 cell lines; the mechanism of action of HDAC2 was found to be enhanced by acetylation of histone H4 bound to the 5-HTT promoter region leading to the expression of 5-HTT by the chromatin immunoprecipitation technique. The expression of 5-HTT correlated with the phenomenon of autophagy in tumor cells, suggesting that HDAC2 plays a role in tumor cell autophagy and apoptosis through the downregulation of 5-HTT expression.

## 2. Materials and Methods

### 2.1. Gene Database

The GEO database (https://www.ncbi.nlm.nih.gov/geo/) provided GSE16011, GSE31262, and GSE90598. DEGs between GBM samples and healthy brain tissue were analyzed using *R* software. Affy *R* tool processed the downloaded raw data, while the limma *R* package identified DEGs. DEGs were discovered using volcano's differential expression volcano charting with |log2FC| 2 and *p*0.01.

### 2.2. Gene Function Analysis

GO and KEGG analyses were performed on genes to determine the enrichment function and the pathway of DEG. The enrichment results were constructed and visualized by the Barplot package. The STRING database (https://string-db.org/) is mainly used for protein interaction network analysis.

### 2.3. Glioma Database

This study employed the TCGA (Cancer Genome Atlas) database to compare HDAC2, DNMT3B, and Bcl2 expression between glioma and normal individuals. The China Glioma Genome Atlas Project (CGGA) database is a user-friendly web tool for studying brain tumor datasets from a Chinese cohort of more than 2,000 samples. The CGGA database analyzed the expression levels of HDAC2, DNMT3B, and Bcl2 in WHO-graded gliomas. The median expression values of each gene in the glioma samples were calculated, and they were classified into high (above median) and low (below median) expression groups. The prognostic results obtained from the CGGA database, including overall survival, were used to plot Kaplan–Meier survival curves, and the relationship between gene expression and HDAC2 and DNMT3B, DNMT3B and Bcl2, and HDAC2 and Bcl2 expression in gliomas established gene correlations.

### 2.4. Statistical Analysis

All experiments were performed in triplicate, and all data are expressed as mean ± standard error (SE). Differences between two groups were analyzed by Student's *t*-test, differences between at least three groups were determined using one-way ANOVA, and results for glioma activity were analyzed using two-way ANOVA. Post hoc analyses were performed after one-way or two-way ANOVA. An SPSS 22.0 for Windows was used to perform these analyses (SPSS, IL, USA), and *P* < 0.05 was considered a significant difference between groups.

## 3. Results and Analysis

### 3.1. Identification of Differentially Expressed DEGs in GBM

Using the GSE16011 dataset, 346 DEGs were upregulated and 241 were downregulated in GBM samples compared to normal human brain tissue (Figure 1(a)). 286 upregulated and 222 downregulated DEGs were found in GSE31262 (Figure 1(b)). 277 upregulated and 162 downregulated DEGs were found in the GSE90598 dataset (Figure 1(c)). 28 genes were co-upregulated and 16 were co-downregulated in the three datasets (Figure 1(d)).

### 3.2. Enrichment Analysis of DEGs

Most of the differential genes in the biological process (BP) category mediated “nervous system development,” “transcriptional regulation,” “DNA replication,” and “apoptosis” (Figure 2(a)). Most differential genes in this category are located in “cytoplasm,” “centrosome,” and “apoptosis” (Figure 2(a)) and “centrosome,” “plasma membrane,” and “cell surface” (Figure 2(b)). Different genes conduct “protein binding,” “transcription factor activity,” “methylation activity,” “transcriptional activity,” and “transcriptional regulatory activity” in the MF category, “Regulatory transcription” (Figure 2(c)). In the KEGG pathway enrichment analysis, we observed that the genes were predominantly enriched in the Wnt pathway (Figure 2(d)). We found that the differential genes in glioma mainly affect the apoptotic process and may influence transcriptional activity and DNA methyl transfer activity.

### 3.3. HDAC2-DNMT3B-Bcl2 Regulation May Occur in Gliomas

The interactions between differential genes were explored, and a PPI network was constructed. With confidence = 0.6, 52 linkages and 38 nodes were found in the network, and the gene axis was observed. We found that DNMT3B has some binding relationship to Bcl2; in the previous GO enrichment analysis, we found that the gene performs a DNA methylation transfer function. In the PPI network, HDAC2-DNMT3B-Bcl2 is the most likely glioma gene axis (Figure 3(a)). Raw signal analysis showed HDAC2 at 329–339 bp on the DNMT3B promoter (Figure 3(b)). In cultured glioma cells T98 G and A172, HDAC2 and DNMT3B binding was confirmed. The ChIP test identified enrichment on DNMT3B promoter, and HDAC2 downregulation dramatically reduced the enrichment of HDAC2 at 329–339 bp, demonstrating that HDAC2 and DNMT3B bind to each other in glioma cells T98 G and A172 (Figure 3(c)). The CpG island of Bcl2 was produced using MethPrimer, positioned at 454–613 bp of the promoter (Figure 3(d)).

HDAC2 was elevated in gliomas, and patients with high HDAC2 expression had a poorer prognosis. We examined the HDAC2 distribution data of WHO patients with different grades from the CGGA database to determine the link between HDAC2 expression and glioma grade (Figure 4(a)). DNMT3B was considerably enhanced in gliomas in the CGGA database, and high expression was related to shorter overall survival in all glioma grades. Bcl2 expression was much lower in gliomas, and low expression was linked to poor patient survival and WHO grade progression (Figure 4(b)). HDAC2-DNMT3B-Bcl2 was positively associated with the glioma database (Figure 4(d)).

## 4. Discussion

The concept of histone acetylation modification was introduced by Vincent et al. [53] back in the 1860s. Histone deacetylases are enzymes that act on histones and related nonhistone proteins and are mainly found on the nucleosomal units that constitute chromosomes; therefore, histone modifications are closely related to gene expression on chromosomes.

Histone acetylation modifications, i.e., entire ATGC order of DNA, alter gene function through structural acetylation modifications of histones. In addition to histone acetylation modification, there are other aspects, such as DNA methylation, chromosome remodeling, noncoding RNA regulation, and genomic imprinting. In this experiment, we focus on histone acetylation; i.e., the transfer and deacylation of acetyl groups. In normal cells, this process is at an emotional level. When stimulated by external factors, such as radiotherapy and chemotherapy in tumor patients, the balance is disturbed, leading to cellular derangement, in which histone deacetylases (HDACs) and histone acetylases (HATs) play an important role.

HDACs [16] de CH3CO- makes histones with corresponding + charge, which has a mutual attraction with DNA(-), making nucleosomes dense and tightly curved and chromosomes in a closed state, which is unfavorable for gene expression; HATs, on the contrary, add acetyl groups to histones with the corresponding (-) charge, which repels DNA(-), making nucleosomes sparse and chromosomes lose, which is favorable for the gene transcription process. Therefore, the imbalance of HDACs and HATs is associated with various gene-related diseases, especially in tumors, as it is closely related to the expression of various oncogenes and oncogenes. Different types of HDACs act at different sites in different cells. Their actions are not random but target specific transcription factors in the nucleus to inhibit the expression of relevant oncogenes, leading to dysregulation of a cycle, proliferation, and differentiation and contributing to tumorigenesis [17].

HDACs act in tumor cells mainly through the following actions: through chromatin remodeling as in acute promyelocytic HDACs act on cycle-related factors, such as the p21 cytokine-dependent kinase inhibitor CDKI class, an important one [18], and class I HDACs are dependent on Sp1/Sp3 to inhibit p21 expression in colon cancer [19, 20]. To ensure accurate entry of cells into the cycle, cells have cycle checkpoints [21], monitoring cells from G1 to S phase or from G2 to M phase. Activating the checkpoint pathway leads to phosphorylation and activation of checkpoint proteins, such as ATR, ATM, CHK1, CHK2, and p51. In addition to phosphorylation, acetylation and deacetylation of cell cycle proteins have a huge impact. HDACs de HDACs are not only associated with the cell cycle but also with apoptosis. HDAC3 in class I HDACs have a clear antiapoptotic effect, and caspase-dependent inactivation of HDAC3 cleavage can activate apoptotic factors and thus trigger apoptosis [22]. In addition to this, HDAC5 in class II HDACs combined with vascular endothelial growth factor (VEGF) is involved in tumor angiogenesis, and the PKD-dependent phosphorylation-specific deletion of HDAC5 inhibits VEGF-mediated expression of an oligomeric nuclear receptor (RN4A1), endothelial cell migration, and angiogenesis in vitro [23]. It can be seen that HDACs are mainly involved in chromatin remodeling, act on cyclin and related apoptotic proteins, and are associated with tumor angiogenesis.

HDACs are closely related to drug resistance in various types of tumor cells. Kikuchi et al. found that the sensitivity of multiple myeloma cells to bortezomib both in vivo and in vitro depended on the expression of HDAC2, implying that HDACs are closely related to proteasome inhibitors. Catley reported that NVP-LAQ824, an inhibitor of HDACs and hydroxamic acid salt derivative, affects proteasome activity in multiple myeloma. This compound uniquely affects multiple myeloma cell adhesion-mediated drug resistance (CAM-DR). It hasa unique effect. Shearer and Saunders [24] found a series of molecules and proteins (p21, CXCR4, syndecan-1, IGF-1, cyclinB2, cyclinF, and Bcl2) were affected by HDACs inhibitors SAHA and bortezomib by the microarray technique. Lung cancer cells also exhibit HDAC activity in resisting cell death through epithelial-mesenchymal transition [23], and many HDAC inhibitors have been widely used in clinical treatment [25]. HDAC2, as part of the transcriptional coblocker complex, is an important and ubiquitous regulator of gene expression. Sheng et al. [26] found that HDAC2 overexpression may induce the proliferation or differentiation of prostate cancer. However, a contrary study found that HDAC2 and suppression of HDAC2 triggered the development of hematological malignancies. This suggests that HDAC2 has a dual identity in tumor development [27]. However, in most classes of tumors, HDAC2 overexpression is a worsening effect on tumors, as in the melatonin treatment study of lung adenocarcinoma [28], where melatonin downregulated HDAC2 expression and led to acetylation of histone H3 in two cell lines, A549 and PC9, and enhanced melatonin-induced apoptosis after the addition of HDAC2 siRNA to bring it down.

We focused on HDAC2 in class I HDACs in the context of glioma drug resistance. Glioma is one of the most difficult tumors to treat, mainly due to its site-specificity and drug resistance [29]. Different individuals have different sensitivity to chemotherapeutic drugs, so finding glioma drug resistance targets is the basis for improving the clinical efficacy of glioma. In our previous study, we screened glioma drug resistance-related genes by gene microarray CHIP and identified 21 differentially expressed genes (including six upregulated genes and 15 downregulated genes); they were related to cell growth and differentiation, apoptosis, and signal transduction, respectively [30], among which HDAC2 was most obviously upregulated. In order to verify the accuracy of the microarray, the gene was confirmed to be highly expressed in drug-resistant gliomas by RT-PCR, so HDAC2 was studied as an important target. HDAC2 is highly expressed in several types of solid tumors, and abnormal expression of HDAC2 [31] can lead to chromosomal structural instability and DNA repair defects, which are associated with the repair of nonhomologous end-joins of broken double strands. HDAC2 expression was found to differ significantly between malignant prostate cancer focal tissue and adjacent benign paracancerous tissue by immunohistochemical staining, revealing that HDAC2 expression differs in similar tumor cells with different degrees of deterioration [32]. Thus, HDAC2 could be a reference indicator for predicting tumor deterioration grade. The HDAC2-DNMT3B-Bcl2 axis in gliomas is differentially expressed and interacting, HDAC2 activates the transcriptional activity of DNMT3B, and DNMT3B inhibits the expression of Bcl2. HDAC2 and DNMT3B are highly expressed in gliomas and have a poor prognosis, while Bcl2 is low expressed in gliomas and has a better prognosis. HDAC2-DNMT3B-Bcl2 promotes Wnt pathway activity in cells and tissues. Low expression of HDAC2 inhibited cell proliferation and migration activity and promoted apoptosis. In contrast, DNMT3B inhibited the downregulation of HDAC2 by increasing cell activity and decreasing apoptosis, and Bcl2 inhibited the effect of DNMT3B to decrease cell activity and increase apoptosis. In vivo, tumorigenic assays showed that HDAC2 downregulation and Bcl2 inhibited tumorigenic activity and enhanced apoptosis in glioma cells, while DNMT3B promoted tumorigenic activity and inhibited apoptosis in tissues.

## Figures and Tables

**Figure 1:** Search for differential genes in GBM. (a) Plotting volcanoes to identify differential genes in GSE16011. (b) Identification of differential genes in GSE31262 dataset. (c) Identification of differential genes in GSE90598. (d) Wayne plot overlap to calculate common upregulated and downregulated genes.

**Figure 2:** Functional enrichment analysis of genes. (a)–(c) GO analysis of genes with the terms biological process, cellular component, and molecular function, respectively. (d) KEGG pathway enrichment analysis of genes.

**Figure 3:** Probe the axis of gene action in GBM. (a) Protein interactions between genes found by STRING. (b) Predicted binding site to HDAC2 on DNMT3B promoter obtained. (c) ChIP experiment to verify the relationship between HDAC2 and DNMT3B. (d) Raw letter analysis to obtain the CpG island of the Bcl2 promoter. (e) ChIP experiment to verify the enrichment of DNMT3B HDAC2-DNMT3B-Bcl2 expression correlates in glioma.

**Figure 4:** Detection of gene prognosis. (a) Detection of TIPARP expression, (b) IFI27 expression, (c) RNF146 expression, and (d) PDE48 expression in GBM.

## Data Availability

The analyzed datasets generated during the study are available from the corresponding author upon request.
